# The Scheme of Ecological Environment Governance under International Discourse Power from the Perspective of Ecological Civilization

**DOI:** 10.1155/2022/3367200

**Published:** 2022-09-20

**Authors:** Zhike Yu

**Affiliations:** Institute of Foreign Language, Jiangxi Science and Technology Normal University, Nanchang, 330000 Jiangxi, China

## Abstract

Ecological civilization construction is an important field of global ecological environment governance, and biodiversity is an important foundation of ecological civilization construction. In the process of building international discourse power of ecological civilization, governments, enterprises, and individuals should attach great importance to ecological environmental protection. Especially in the context of the new era, the promotion of international discourse power of ecological civilization and the governance of ecological and environmental problems must be in the process of further consolidating the foundation of ecological economy, paying particular attention to the management of enterprise ecological and environmental costs. Therefore, from the perspective of practical research, fuzzy analytic hierarchy process is used to comprehensively evaluate enterprise environmental cost management. Through research, the importance of enterprise environmental cost management and the help to ecological environment management are proved, and on this basis, ecological environment management countermeasures are put forward.

## 1. Introduction

In recent years, with the deepening of China's reform and opening-up policy, China's economy has developed rapidly, and at the same time, China's position in the world economic pattern is becoming more and more obvious. However, with the development of global economy and the rise of China's economic strength, the ecological environment governance issues became the primary problem we must pay attention to, such as air pollution, water pollution, land desertification, and other environmental issues more and more obvious, all these problems hinder our country to build more good ecological civilization is the international voice of important factor. Of course the emergence of these problems and industrial production, economic development has a direct relationship. In particular, the production and sales of industrial enterprises are one of the important causes of these pollutions. Therefore, from the perspective of ecological environmental governance and the construction of international discourse power of ecological civilization, this essay focuses on high-pollution enterprises and takes the construction of ecological civilization as the guide to deeply analyze the importance of ecological environmental cost management in the process of enterprise operation. See Figure 1.

## 2. Literature Review

In western society, human development, and natural environment is so brazenly and its common belief of Christianity has a lot to do—in congregational Christian, god created everything and finally, creates the human, god created everything is for the service of humanity, all things if not for human use, it has no value. It is obvious that this religious axiom will directly lead to the spread of anthropocentrism [1]. Therefore, in order to deal with this problem, American scholars proposed in the middle and late 1960s that ecological problems could not be solved if westerners could not reject the Christian axiom that “nature has no value of existence except for serving human beings”. Some scholars sounded the horn against anthropocentrism for the first time, and it was also during this period that western ecological theories began to form a certain philosophical system, with various schools of thought arguing, including ecocentrism, ecological Marxism, modern anthropocentrism, ecological politics, and ecological ethics [2].

Some scholars especially emphasized the important role of cultural identity in the world order. He divided the world into eight civilizations and believed that after the disintegration of the bipolar structure, the clash of civilizations would become more significant. From the perspective of discourse power, culture is an important way to enhance discourse power. We should not only respect the differences between different cultures but also actively seek commonalities, enhance exchanges, and build a new type of international relations. Similarly, some scholars put forward the concept of “soft power”; that is, in addition to hard power such as military and economic power, cultural and political values, and the ability to make rules and decide political issues in the international community, which indicates that the power of discourse is not only reflected in some material levels but also in many abstract levels [3]. The above views have important implications for the research on the promotion of discourse power.

The research on the theoretical basis of discourse power of ecological civilization in China is the starting point for the study of discourse power of ecological civilization [4]. Some scholars believe that today's China has enough confidence in discourse. It is pointed out that the discourse confidence of China's ecological civilization construction comes from the common value appeal of mankind, the profound traditional Chinese ecological wisdom, the rich practice of ecological civilization construction, and the moral power of China's ecological civilization construction. Therefore, in the process of building the discourse system of China's ecological civilization construction, it is necessary to get rid of discourse dependence and discourse worship on the West, break through the “discourse deficit”, strengthen discourse confidence in China's ecological civilization construction, and strive for international discourse power [5]. Some scholars from the perspective of system confidence argue that China improve the influence condition of ecological civilization, if it is thought that the Chinese voice to promote ecological civilization have superior socialist system as the backing, has high efficiency of system effectiveness for the reality basis, and has a profound experience and abundant practical results for history basis, a system of deep popularity for value basis. Therefore, the conditions for the promotion of discourse power are relatively mature [6]. Some scholars view it from the perspective of the challenges faced by the discourse power construction of China's ecological civilization. For example, under the traditional international discourse system of “the west is strong and the east is weak”, some media and scholars in the western society wear colored glasses, ignoring our achievements in the construction of ecological civilization; we amplify and spread some existing environmental problems [7].

## 3. Current Situation and Problems of Ecoenvironmental Cost Management of Enterprises in China

### 3.1. General Situation of China's Industrial “Three Wastes” Discharge

1. Total emission of industrial pollution and its increase and decrease in China

First, analyze waste water discharge. As can be seen from Table 1 and Figure 2, since 2004, with the improvement of industrialization and urbanization, the national wastewater discharge has been increasing. In 2014, wastewater discharge exceeded 70 billion, reaching 71.62 billion tons. Compared with 2004, the increase was 23.38 billion tons, an increase of 48.47%, with a large increase. Among them, industrial waste water emissions were generally flat, reaching a peak of 24.66 billion tons in 2007, and then, gradually decreased. From 2006 to 2010, the national wastewater discharge increased steadily with a small increase, in which the industrial wastewater discharge was basically flat, and the increase or decrease ratio was controlled within 3%. From 2011 to 2014, the country's wastewater emissions increased by 5.7 billion tons, up 8.65 percent year on year, while industrial wastewater emissions decreased by 2.56 billion tons, down 11.09 percent year on year. From Figure 2, it is obvious that the “scissors difference” between national wastewater discharge and industrial wastewater discharge increases gradually.

Figure 3 shows that in 2004–2005, the growth rate of sulfur dioxide industry was 14.6% and the growth rate of smoke and dust was 3.8%. During November five year, industrial sulfur dioxide emissions, industrial fumes and dust emissions showed a downward trend, with a decrease rate of 16.68% and 37.12%, respectively, exceeding the emission reduction target. Only industrial nitrogen oxide emissions and growth rates were on the rise, and the increase was significant in the last year, reaching 14.1% month-on-month, an increase of 11.4 percentage points compared with 2009. After 2011, except for industrial smoke and dust, which rose sharply in 2014, all three kinds of pollutants have declined at different ranges [8].

As can be seen from Figure 4, the industrial solid waste increased year by year from 2004, with a fast growth rate. In 2010, the growth peaked in 2011. The sequential growth rate in 2011 was as high as 34%, and the total annual production was basically flat after that. It can be seen that Chinese enterprises need to further improve their emission control and emission standards for solid waste [9].

(2) Overview of investment in environmental pollution control

As can be seen from Figure 5, China's investment in environmental pollution control has been increasing steadily since 2004, and exceeded 700 billion yuan in 2010 and reached 951.65 billion yuan in 2013, showing an overall upward trend. It can be seen that China is highly concerned about environmental problems and has taken actions to invest in and improve environmental pollution control on a large scale. From the analysis of the total amount of waste water and other pollutants discharged and the general situation of increase and decrease, it can be seen that China's control of pollution discharge is slightly effective. However, China's investment in industrial pollution control has not increased, accounting for less than 10%, and the relative investment proportion has even decreased [10].

### 3.2. Construction of Enterprise Ecoenvironmental Cost Management Evaluation Model

In this study, the fuzzy analytic hierarchy process (FAHP) combined with the two methods is used to comprehensively evaluate the environmental cost management system. According to “resource saving and protection” and “environmental protection and management” in the path of ecological civilization construction, the resource benefit index and environmental benefit index are put forward, and the economic benefit index and social benefit index are put forward according to the economic development and external social image of enterprises. These four indicators are used to evaluate environmental cost management [11]. The environmental cost management evaluation system adopted in this paper is shown in Figure 6:

#### 3.2.1. Determine Index Weight

This study used the unambiguous analytical hierarchical (FAHP) technique to determine the weight of each measure. The fuzzy analysis hierarchy (FAHP) receives the fuzzy filtering matrix by comparing the tests, and finally, obtains the weight of each instrument through the fuzzy filtering matrix.

Due to the influence of each indicator at the subindicator level on the indicator level and the influence of each indicator at the target level are not the same, the importance of each indicator at the upper level is also different. In the analytic hierarchy process, pairwise comparison is carried out on each indicator in the subindicator layer and indicator layer to judge the importance, and the relevant fuzzy judgment matrix is finally obtained by using the 1-9 scaling method as shown below [12], as shown in Table 2.

A hierarchical scale is the weight of the sequence of values of the index process obtained by counting the unknown filtering matrix to the next target layer. The special steps are as follows.

Firstly, the product of each row of elements of the fuzzy judgment matrix needs to be calculated, as

(1) $$\begin{array}{c} M_{i}=\overset{n}{\underset{j=1}{\prod }}a_{ij},i=1,2,\cdots ,n. \end{array}$$

Calculate the NTH root of *M*_*i*_, as

(2) $$\begin{array}{c} {\bar{W}}_{i}=\sqrt[{n}]{M_{i}}. \end{array}$$

Secondly, the vector (Equation (3)) is normalized to obtain Equation (4):

(3) $$\begin{array}{c} \bar{W}={\left({\bar{W}}_{1}\;{\bar{W}}_{2}\;\cdots \;{\bar{W}}_{n}\right)}^{T}, \end{array}$$

(4) $$\begin{array}{c} W_{i}=\frac{{\bar{W}}_{i}}{\sum_{j=1}^{n}{\bar{W}}_{j}}. \end{array}$$

Formula (5) is the eigenvector of index weight obtained.

(5) $$\begin{array}{c} W={\left(\begin{array}{cccc} W_{1} & W_{2} & \cdots & W_{n} \end{array}\right)}^{T}. \end{array}$$

Then, calculate the maximum characteristic root of the fuzzy judgment matrix, as

(6) $$\begin{array}{c} \lambda_{\max}=\overset{n}{\underset{i=1}{\sum }}\frac{{\left(AW\right)}_{i}}{{nW}_{i}}, \end{array}$$

where (*AW*)_*i*_ represents the *i* element of vector*AW* .

#### 3.2.2. Consistency test

The consistency index is calculated, as

(7) $$\begin{array}{c} CI=\frac{\lambda_{\max}-n}{n-1}. \end{array}$$

The magnitude of the measured value indicates the difference in resolution of the filter matrix. The lower the measurement value, the better the consistency of the filter matrix. It indicates the value of the mean of the relative mean of the unknown visible matrix, as shown in Table 3.

Because the first and second order judgment matrices are definitely identical, there is no need to test, and *RI* is always 0. When the order of the judgment matrix is ≥3, the random consistency ratio (CR) can be calculated to determine whether the judgment matrix has satisfactory consistency, as

(8) $$\begin{array}{c} CR=\frac{CI}{RI}, \end{array}$$

when *CR* < 0.10, the judgment matrix has satisfactory consistency. If not, it is necessary to correct the judgment matrix to make it have satisfactory consistency. Therefore, the importance measurement of each expert on each evaluation factor, namely weight, can be finally determined, and the follow-up judgment can be made according to the weight (*W*).

### 3.3. Steps of Environmental Cost Management Evaluation

1. To establish the target enterprise environmental cost management evaluation system
2. To determine the fuzzy comprehensive evaluation set

The fuzzy comprehensive evaluation index factor set as

(9) $$\begin{array}{c} U_{i}=\left(\begin{array}{cccc} U_{1} & U_{2} & \begin{array}{cc} U_{3} & \cdots \end{array} & U_{m} \end{array}\right). \end{array}$$

The evaluation index factor set is subdivided into *N* evaluation subindex factor sets according to index attributes,

(10) $$\begin{array}{c} U_{i}=\left(\begin{array}{cccc} U_{i1} & U_{i2} & \begin{array}{cc} U_{i3} & \cdots \end{array} & U_{i,j} \end{array}\right),i=1,2,3,\cdots ,m;j=1,2,3,\cdots ,n. \end{array}$$

*M* = 4 in the comprehensive evaluation model in this paper, where

(11) $$\begin{array}{c} U=\left\{\begin{array}{cccc} U_{1} & U_{2} & U_{3} & U_{4} \end{array}\right\}=\left\{\text{Environmental benefits},\text{Environmental benefit},\text{Economic benefits}\right\},\\ U_{1}=\left\{\begin{array}{cccc} U_{11} & U_{12} & U_{13} & U_{14} \end{array}\right\},\\ U_{2}=\left\{U_{21},U_{22},U_{23}\right\}=\left\{\text{Conservation of hydropower resources}\right\}. \end{array}$$

To set up comments and values, this evaluation model defines the comment set as

(12) $$\begin{array}{c} V=\left\{V_{1},V_{2},V_{3},V_{4},V_{5}\right\}=\left\{\text{Good},\text{Medium}\right\}. \end{array}$$

The evaluation value set is shown in

(13) $$\begin{array}{c} \left\{100,80,60,40,20\right\}. \end{array}$$

According to the comprehensive research and analysis of invited experts, each index is evaluated and scored to achieve qualitative and quantitative transformation. Meanwhile, according to the membership degree of each index, the fuzzy evaluation matrix *R* of each evaluation factor of the secondary index and the main index is finally obtained [13]. The determination of membership degree is a key step in the application of fuzzy mathematics. The determination of membership degree is a key step in the application of fuzzy mathematics. However, because the whole process depends on human subjectivity, this paper introduces trigonometric fuzzy function to determine feasible relative index membership degree, as

(14) $$\begin{array}{c} R_{ij}=\left(\begin{array}{c} R_{i1}\\ R_{i2}\\ \cdots \\ R_{ij} \end{array}\right). \end{array}$$

The weight matrix *W*_*i*_ of the secondary index obtained above and the fuzzy evaluation matrix *R* of the first-level fuzzy comprehensive evaluation determined by the membership function of the previous step are combined to obtain the first-level fuzzy comprehensive evaluation, as

(15) $$\begin{array}{c} B_{i}=W_{i}*R_{i},i=1,2,3,4. \end{array}$$

From the four benefit indicators to the target company's “environmental cost management” final comprehensive evaluation. In other words, the second-level comprehensive evaluation results can be obtained by multiplying the fuzzy evaluation matrix *R* composed of the weight *W* of each index at the index layer and the evaluation results of each index at the index layer, as

(16) $$\begin{array}{c} B=W*R=W*\left(\begin{array}{c} B_{1}\\ B_{2}\\ B_{3}\\ B_{4} \end{array}\right). \end{array}$$

The final result score of *E* is the comprehensive evaluation of the environmental cost management of the target company. The score of *E* is obtained by multiplying the comprehensive evaluation value of the target layer and the evaluation value set, as

(17) $$\begin{array}{c} E=B*V^{T}. \end{array}$$

The higher the value of *E* is, the better the target company performs in environmental cost management and the higher its environmental performance is; otherwise, the worse.

### 3.4. Evaluation of XY Company's Environmental Cost Management from the Perspective of Ecological Civilization

#### 3.4.1. To determine Index Weight

In order to ensure the effectiveness and completeness of expert management evaluation, XY Steel Company invited 10 experts in related professional fields and set up a management evaluation group. The specific results are shown in Tables 4–9.

From Table 9, we can intuitively see the degree of influence of the subindicator layer on the main indicator layer and the main indicator layer on the target layer [14]. For example, in the evaluation of environmental cost management of XY Iron and Steel Company, environmental benefit index, and economic benefit index are equally important, and resource benefit is in the second place. Therefore, the current environmental problems are serious; all walks of life should give high attention. As for environmental benefit indicators, the expert group believes that environmental protection is very important in advance, while carbon transaction costs/benefits and pollutant and waste treatment rates are relatively less important. As for the resource benefit index, the comprehensive utilization of materials is very important, and the conservation of hydropower resources and waste reuse are at a slightly important level. As for economic benefit index, the importance of environmental investment return on capital is 0.4258, which is in an important position. For social benefit indicators, a good and positive image of environmental protection is very important [14].

On this basis, combined with the above series of formulas, the following results can be obtained through calculation, as shown in Table 10:

It can be seen that the comprehensive evaluation result of environmental cost management of XY Iron and Steel Company is 76.9127, which is above the middle level. Environmental benefit and resource benefit are also close to good level. This shows that XY Steel Company has paid great attention to environmental pollution and resource shortage, and relevant environmental protection measures and actions have achieved initial results [15]. As for economic benefits, in recent years, the world economy continues to operate at a low level, while China's economy develops slowly and its growth rate continues to shrink, leading to oversupply in the steel market, increasingly intensified homogeneous competition, and relative decline in economic benefits. Therefore, the economic benefits of XY Steel Company are at an above medium level. As for social benefits, XY Steel Company, as the industry leader, needs to invest more in corporate environmental protection and product environmental protection. The increase of costs will affect corporate profits, and the contradiction between the two also makes the social benefits of the company at an above medium level.

## 4. Governance Countermeasures under International Discourse Power of Ecological Environment

### 4.1. To Improve Government Ecological and Environmental Governance

1. To establish the government's responsibility for ecological and environmental governance

First of all, the government has the responsibility to protect the natural ecological environment. Natural environment is the fundamental environment for human survival, the premise for human production and life, and the fundamental place for human survival [16]. However, in the process of human development, there are many phenomena that destroy the natural ecological environment, which seriously affect human survival and development. Some human behaviors seriously damage the natural ecosystem and break the balance of the ecosystem. These behaviors will eventually lead to the destruction of human living environment. The government, as an institution to safeguard the survival and development of human beings, has the obligation to take on the responsibility of protecting the living environment of human beings, and at the same time has the responsibility to punish and supervise the destruction of the natural environment.

Second, the government has an obligation to avoid ecological damage caused by market imbalances. The market has a direct impact on the ecological environment. Market failure is a potential threat to the ecological environment, so it is the duty of the government to maintain the orderly market and ensure the standardization of the market. We will strengthen oversight and management of the market to ensure that it operates in an orderly manner and does not threaten or damage the ecological environment. Collectives and individuals who violate market rules and cause environmental damage shall be punished to make violators pay the price, increase the cost of violation, and make the behavior of destroying the ecological environment pay the due price.

(2) Government ecological environment administrative responsibility type

Subjective administrative responsibility refers to the subjective administrative feeling of government administrative staff, the conscience and loyalty of administrative staff, and the subjective initiative and autonomy of administrative staff. The realization of administrative responsibility depends on the subjective consciousness of administrators. Therefore, the government's environmental subjective administrative responsibility depends on the government staff's subjective consciousness of environmental responsibility, and the government's environmental subjective administrative responsibility is a subjective feeling, conscious recognition, and active practice of the government administrator. The subjective environmental administrative responsibility of the government is gradually produced in the process of human socialization, and is an indispensable part of the process of human environmental protection [17]. In the process of carrying out the environmental administrative responsibility, the government cannot lack the subjective administrative responsibility of the government. The subjective administrative responsibility of the government is of great significance for the government administrators to deal with various environmental responsibility problems.

Objective administrative responsibility refers to the responsibility delivered by laws, regulations or administrative personnel. Therefore, the objective administrative responsibility of the government ecological environment refers to the ecological environment management and protection responsibilities that the government administrators should do according to laws and regulations or entrusted by the superior.

### 4.2. To Improve the Rule of Law for Government Ecological and Environmental Management

1. To promote reform of the government's judicial system for ecological and environmental protection

First, try to handle cases in different places of the judicial system to avoid excessive interest involvement of the judicial organ in the region and improve the independence of handling cases [18]. Second, in terms of funds, the central government can be used to allocate funds to solve the problem that judicial institutions are subject to local governments in terms of financial power. Third, we should strengthen supervision over the effectiveness of judicial organs in enforcing the law and strengthen their functions in ecological and environmental governance. Fourth, “third party forces” such as the public and social groups should be given the right to file ecoenvironmental lawsuits to ensure that the public and social groups have the right to supervise the behavior of destroying the ecological environment or the absence of functions of government agencies [19]. Fifth, it is necessary to establish and improve the internal supervision mechanism of judicial organs, crack down on judicial corruption, and build a clean and efficient judicial team [20].

(2) To improve government law enforcement of ecological and environmental issues

On the premise of “there are laws to abide by and to be observed”, we should also ensure that “there are laws to be observed, law enforcement is strictly enforced and lawbreakers are prosecuted”. For ecological environmental governance, while ensuring the integrity of laws and regulations related to the ecological environment, we should also improve the level and efficiency of law enforcement of ecological environmental governance. Specifically, the following points should be done: first, education and training activities should be carried out to educate and study law enforcement teams on national laws, regulations, guidelines, and policies, so as to improve the level of law enforcement and ensure that law enforcement conforms to national laws and regulations. Second, we should promote the anticorruption work of the ecological environment law enforcement team, resolutely crack down on the rent-seeking behavior of the ecological environment law enforcement officers, and strictly punish the corrupt behavior to ensure the integrity of the ecological environment law enforcement team [21].

## 5. The Practical Path to Enhance the Discourse Power of Ecological Civilization in China in the New Era

### 5.1. Actively Build China's Discourse System of Ecological Civilization

1. To make full use of the rich local ecological and cultural resources

The construction of discourse system of ecological civilization in China must be based on the rich local ecological and cultural resources, based on China's historical practice, and combined with the current development needs, so as to make this system have a solid foundation [22]. In order to meet the needs of the current construction of ecological civilization, we can completely absorb nutrients from traditional culture to innovate the theory of ecological civilization in our country and strengthen the discourse right of ecological civilization in our country. For example, the ancients advocated thrift, opposed extravagance and waste, and moderately took from and enjoyed from nature, rather than burning forests and farmland or draining water and fishing, so as to achieve the coordination between man and nature [23]. This idea can be used to counter the increasingly serious consumerism in the market economy and alleviate the current situation of valuing consumption and economic development rather than human beings themselves. Actively innovating China's ecological civilization thought through China's local cultural resources is the embodiment of “cultural confidence”, which is not only of realistic significance to the present but also of great significance to the Sinicization of Marxist theory [24].

(2) To fully excavate Marxist classical ecological discourse

The situation of ecological civilization in today's world is complicated and more complicated. It is beneficial to solve the problem and establish the discourse system of ecological civilization to make Marx's classical theory adapt to the development status of human society through innovative elaboration and explanation. In fact, many thoughts and concepts of ecological civilization in China are influenced by the classical ecological discourse of Marxism, such as “people-oriented” and “harmonious society” advocated by the “Scientific Development Concept”, “clear water and green mountains are gold and silver mountains” proposed by General Secretary Xi Jinping, and “ecological prosperity leads to civilization prosperity”. Besides, the viewpoints of “ecological decline means civilization decline” and “life community” excavate the classical ecological discourse of Marxism to varying degrees. Of course, Marxist thought still has a strong time; many theories still need to be combined with the needs of the reality to explore, so as to further use.

### 5.2. To Condense and Sublimate Chinese Ecological Civilization Theory Achievement and Experience Summary

The theoretical achievements and experience summary of China's ecological civilization is based on the practical experience of the Chinese people's ecological civilization construction led by the party and state leaders since the founding of the People's Republic of China 70 years ago, especially since the reform and opening up, which has made the theory and practice of ecological civilization from scratch, from weak to strong, and finally, achieved today's brilliant achievements. In order to construct the discourse system of ecological civilization in China, it is necessary to further condense and sublimate the theoretical achievements and experience summary of ecological civilization in China. Practice is the basis of cognition and the only standard to test the truth. The theoretical achievements and practical experience of China's ecological civilization construction are the most solid foundation for the construction of discourse system.

The historical experience of China's splendid achievements in ecological civilization can be summarized as follows: first, the construction of ecological civilization adheres to the leadership of the Communist Party of China (CPC), which is the only political force in China with overall planning. The overall planning of ecological civilization, the formulation of laws, and the tackling of difficulties are inseparable from the role of the Party. The leadership of the Party is the political guarantee of ecological civilization construction. Second, we need to put the people first. The people are the creators of history. We need to mobilize the enthusiasm of the people in our efforts to promote ecological progress. Third, we need to rely on system construction to ensure the effective progress of ecological civilization construction. We need to analyze specific problems on a case-by-case basis, formulate laws and regulations according to local conditions, and ensure that law enforcement is strictly enforced and violations of laws are prosecuted. Finally, we should pay attention to the combination of ecological civilization construction and economic development, avoid “campaign-style” governance, give overall consideration to environmental protection and economy, and formulate different laws and regulations in different historical periods to meet the needs of the times.

### 5.3. To Expand External Exchanges of Ecological Progress

1. To use the communication power of we media to construct a kind of green values

As a socialist country, it should learn to use the basic principles of Marxism as a weapon, in line with the concept of “a community with a shared future for mankind”, and use the communication power of we media to promote the construction of a novel international ecological governance values. This kind of values should make people realize that the fate of the earth is closely related to everyone, and infinite expansion of individualism will lead to disaster. Therefore, it is necessary to make a thorough change to the original life and actively establish a green and sustainable new way of life.

(2) To attach importance to the construction of overseas online media platforms

Some traditional Chinese media should pay more attention to the construction of overseas online media platforms, and some well-known employees of propaganda agencies should also actively participate in overseas new media platforms to interact with foreign netizens by answering questions to narrow the distance, and show a good image of China to the world. In addition, in the era of the media, information spreads rapidly, so it is more important to actively seize the right to speak. Environmental pollution is an inevitable phenomenon in the development process of any country. In the face of negative events, including ecological problems, if the government hides it, it will be easy to ferment once spread abroad, resulting in widespread rumors, and even become the material for western media to smear China. Therefore, we should try not to hide or cover up the facts, but take the initiative to report the facts, actively seize the right to speak, and demonstrate the confidence of a major country.

## 6. Conclusion

The significance of discourse power of ecological civilization is not limited to the field of ecological environment itself but to meet the needs of China's future development, become a modern socialist power and realize the rise of the Chinese nation. As a traditional weakness in China's development process, on the one hand, it does face a lot of development resistance, and we still need to accumulate experience. At the same time, however, we should be optimistic that after decades of “hiding its strength and biding its time”, the “hard power” that China has accumulated has brought it closer than ever to becoming a power of discourse in ecological civilization, and we should make full use of this opportunity. In view of the analyzed opportunities and challenges, we should enhance the discourse power of ecological civilization from three aspects: the construction of ecological civilization itself, the construction of discourse system of ecological civilization, and the strategy of external communication. Of course, it must also be recognized that the issue of discourse power is a relatively new research topic in China, and the research in the field of discourse power of ecological civilization is relatively rare. Therefore, it is relatively difficult to collect literature in the writing process, and the collected information is not rich enough. In the end, the author only made a slight expansion of the research field on this basis, but in the research process, we can obviously perceive that this is still a field worthy of further research, and hope that the majority of scholars can continue to study.

## Figures and Tables

**Figure 1:** The ecological environment under the international discourse power from the perspective of ecological civilization.

**Figure 2:** Interannual comparison of national wastewater and industrial wastewater discharge.

**Figure 3:** Interannual variation of main pollutants in exhaust gas.

**Figure 4:** Interannual variation of industrial solid waste output.

**Figure 5:** Annual changes in environmental investment pollution control and pollution reduction.

**Figure 6:** Evaluation model of enterprise environmental cost management from the perspective of ecological civilization.

**Table 1:** Overview of pollution emission and its increase and decrease in China.

	National waste water		Industrial waste water		Industrial sulfur dioxide		Industrial nitrogen oxide		Industrial smoke and dust		Industrial solid waste	
	Total emissions (tons)	Sequential growth (%)	Total emissions (tons)	Sequential growth (%)	Total emissions (tons)	Sequential growth (%)	Total emissions (tons)	Sequential growth (%)	Total emissions (tons)	Sequential growth (%)	Total emissions (tons)	Sequential growth (%)
2004	482.4	4.9	221.8	4.5	1891.4	5.6			1791.3	-4.1	12	20.2
2005	524.5	8.7	241.2	10.0	2168.2	14.6			1860.1	3.8	13.4	11.7
2006	536.8	3.2	321.2	1.2	2337.6	3.2			1236.8	-10.1	15.2	13.5
2007	556.8	3.5	246.3	2.7	2140	-4.4	1361.3	11.0	1698.2	-12.1	16.7	15.4
2008	576.5	2.7	241.7	-2.0	1991.0	-6.9	1250.5	-0.9	1526.2	-14.6	10.9	8.0
2009	590.2	2.8	234.8	-3.2	1865.9	-6.3	1284.8	2.7	1280	-10.2	20.4	7.4
2010	617.3	4.7	237.5	-1.2	1685.4	-0.1	1463.1	14.2	1051.9	-6.7	24.1	18.1
2011	659.3	6.8	232.5	-3.1	2017.2	8.2	1789.2	18.0	1100.8	4.7	32.3	34.0
2012	687.1	3.6	221.6	-4.0	1911.7	-5.2	1685.1	-4.1	1029.3	-6.5	32.8	-0.3
2013	698.5	1.5	206.6	-4.0	1835.2	-4.0	1516.5	-6.8	1094.6	6.3	32.6	-0.6
2014	716.8	3.0	201.3	-2.0	1750.4	-5.2	1401.8	-9.1	1546.1	33.0	20.1	0.7

**Table 2:** Significance scale of fuzzy judgment matrix and its meaning.

The serial number	Importance level	*U_ij_* assignment
1	*i* element, *j* element with equal importance	1
2	The *i* element is slightly more important than the *j* element.	3
3	*The i* element is obviously more important than the *j* element.	5
4	The *i* element is stronger than the *j* element.	7
5	The *i* element is extremely more important than the *j* element.	8
6	The *i* element is slightly less important than the *j* element.	1/3
7	The *i* element is obviously less important than the *j* element.	1/5
8	*i* element is strongly not important than *j* element.	1/7
9	Element *i* is extremely less important than element *j*.	1/9
10	Comparison of the importance of elements *i* and *j* between intermediate and adjacent judgment values (qualitative analysis to judge)	2, 4, 6, 8, 1/2, 1/4, 1/6, 1/8

**Table 3:** Average random consistency index.

1	2	3	4	5	6	7	8	9
0.00	0.00	0.45	0.90	1.20	1.24	1.32	1.42	1.44

**Table 4:** Judgment matrix and weight comparison—environmental cost management.

	*U*_1_	*U*_2_	*U*_3_	*U*_4_	The weight(W_i_)
*U*_1_	1	1	1	1	0.2463
*U*_2_	1	1	1	2	0.2849
*U*_3_	1	1	1	1	0.2463
*U*_4_	1/2	1	1/2	1	0.1750

Note: Consistency test : *λ*max = 4.0606, CI = 0.0202, RI = 0.9, CR = 0.0224 < 0.1, meet the requirements.

**Table 5:** Judgment matrix and weight comparison—environmental benefit index.

	*U*_11_	*U*_12_	*U*_13_	*U*_14_	The weight(W_1*j*_)
*U*_11_	1	3	3	3	0.4950
*U*_12_	1/3	1	1/2	2	0.1328
*U*_13_	1/3	2	1	1	0.1996
*U*_14_	1/3	1	1	3	0.1835

Note: Consistency test : *λ*max = 4.0606, CI = 0.0202, RI = 0.9, CR = 0.0224 < 0.1, meet the requirements.

**Table 6:** Judgment matrix and weight comparison—resource benefit index.

	*U*_21_	*U*_22_	*U*_23_	The weight(W_2*j*_)
*U*_21_	1	1/2	3	0.4950
*U*_22_	1/2	1	1	0.4126
*U*_23_	1	1	1	0.3276

Note: Consistency test : *λ*max = 4.0606, CI = 0.0202, RI = 0.9, CR = 0.0224 < 0.1, meet the requirements.

**Table 7:** Judgment matrix and weight comparison—economic benefit index.

	*U*_31_	*U*_32_	*U*_33_	*U*_34_	The weight(W_3*j*_)
*U*_31_	1	2	2	3	0.4950
*U*_32_	1/2	1	2	1	0.2314
*U*_33_	1/3	1/2	1	1	0.1484
*U*_34_	1/2	1	2	2	0.2354

Note: Consistency test : *λ*max = 4.0606, CI = 0.0202, RI = 0.9, CR = 0.0224 < 0.1, meet the requirements.

**Table 8:** Judgment matrix and weight comparison—social benefit index.

	*U*_41_	*U*_42_	The weight(W_4*j*_)
*U*_41_	1	2	0.6667
*U*_42_	1/2	2	03232

Note: Consistency test:*λ*max =4.0606, CI =0.0202, RI =0.9, CR =0.0224<0.1, meet the requirements.

**Table 9:** Weight comparison of primary and secondary indicators on environmental cost management evaluation.

	The main indicators	Time indicators	The weight(W)
Environmental cost assessment management	Environmental benefit index	Ex ante environmental cost	0.4950
		Carbon trading costs/benefits	0.1450
		Treatment rate of pollutants and wastes	0.9968
		Postcontamination treatment	0.1560
	Resource efficiency indicator	Conservation of hydropower resources	0.2599
		Comprehensive utilization of materials	0.4128
		Waste reuse	0.3276
	Economic benefit index	Return on capital for environmental investment	0.4258
		Environmental cost input ratio	0.2312
		Environmental loss cost rate	0.1484
		Environmental restoration cost rate	0.1945
	Social benefit index	Corporate environmental image	0.6667
		Product environmental image	0.2323

**Table 10:** Comprehensive evaluation results of environmental cost management and main indicators.

Project	Environmental cost management	Environmental benefits	Resource efficiency	Economic benefits	Social benefits
Comprehensive evaluation value	76.9125	75.7588	78.7588	75.9982	78.6333

## Data Availability

The labeled data set used to support the findings of this study is available from the corresponding author upon request.
